The article "Design and Research of VR Basketball Teaching System Based on Embedded Intelligent Sensor" was published in 2022. Journal: J Environ Public Health.

# Design and Research of VR Basketball Teaching System Based on Embedded Intelligent Sensor

**DOI:** 10.1155/2022/3688596

**Published:** 2022-07-31

**Authors:** Jinxin Jiang, Shoujiang Wu, Siyu Zhang

**Affiliations:** Department of Physical Education, Bozhou University, Bozhou 236800, Anhui, China

## Abstract

Physical education pedagogy serves as a carrier of physical education theory and practical activities and plays an important role in physical education. The reform and development of education are always related closely to the growth of scientific and technological development, and people's physical education training methods are also undergoing subtle changes. The traditional single and formulaic training methods in the past have gradually turned to modern training methods with better interaction and visibility. All of this prompts people to have new requirements on sports training concepts and training modes. On this basis, teachers can conduct virtual teaching in a more interactive, more involved, and orderly manner in the virtual classroom. This paper constructs the implementation framework of VR basketball teaching auxiliary training, divides students into an experimental group and a control group and tests the physical fitness of students before and after the experiment. The students' basic basketball skills were tested by using embedded intelligent sensors to recognize the students' movements. The experimental results showed that after the test, the four basic basketball skills scores of the students in the experimental group were 68.78, 74.02, 73.13, and 72.34, respectively. The virtual reality basketball teaching system designed in this paper can effectively improve the basketball level of students.

## 1. Introduction

Through the comprehensive adoption of nuclear simulation technology and sports practice, students can obtain intuitive and realistic training effects, thus improving their training awareness and creativity. It has given a positive impetus to the research and innovation of sports training modes. However, since sports training is very different from ordinary physical education, how to make good sense of statistical simulation technology and build a new statistical training model, so as to let students learn and master sports technology more quickly, steadily, and intuitively, is a very meaningful topic.

Regarding basketball teaching, relevant scientists have done the following research. Wang et al. proposed a design optimizing approach for basketball classes and a motion recording technology-based practice system. By making a comparison between the results of the simulation and the real athletes' training videos, a training screen and standard movements are displayed on one screen, and the movements are compared and evaluated [1]. Yan presented relevant research findings and recommendations for the use of multimedia animations in the teaching of basketball tactics. The study demonstrated students' knowledge and skills. He studied the impact of multimedia learning on basketball tactics. A number of objective factors have limited the use of multimedia teaching methods by teachers [2]. Qiu and Zhang studied the development of basketball and the system of computer-based training. By collecting and analyzing three-dimensional data on basketball technology, it is convenient for teachers to continuously integrate and use teaching aids and create an animated database that meets their learning needs. Motion capture technology can be used for parameter analysis and motion analysis, making the teaching process more intuitive and intelligent [3]. Based on video image processing technology, Lv et al. have built a college basketball teaching assistant training system. According to the students' technical movements and related parameters, the training is guided, which effectively solves the shortcomings of the college basketball teaching auxiliary training system and helps improve basketball education [4]. Wang et al. analyzed the application of network resources and digital platforms in college basketball teaching innovation. The basketball teaching network digital resource platform is an open platform resource, which not only has the function of web browsing but also has the function of basketball knowledge learning, which can be used as a reasonable combination of teaching resources [5]. Masadis used three different methods to explore the acceptance satisfaction of primary school students participating in physical education courses, especially the basketball skills teaching process. Teaching methods are a factor in the differentiation of satisfaction; student-centered teaching methods help maximize satisfaction. Gender is not a factor in the diversity of student satisfaction [6]. The main problem of these studies is that they cannot test the teaching effect well.

The main research results for embedded smart sensors are as follows. Ali and Alshmrany proposed an automated plant irrigation system that embeds a smart sensor system and internet of things (IoT) to monitor and manage farms, automatically supplying water to plants and keeping them updated by generating messages. To control these parameters via IoT, the system connects remote devices by connecting the sensor system with a microcontroller [7]. Pham et al. proposed a smart rock embedded with piezoelectric sensors to monitor the electromechanical resistance of concrete damage in the area of the prestressed anchors. Internal damage to the concrete was successfully detected by integrated smart stones, which allowed the technology to be applied to monitor the health of the anchor [8]. Ibrahim et al. examined the limitations of commonly used sensor accuracy and proposed a new error model for the smart device accelerator, which also includes traditional noise as well as the sampling time uncertainty error represented by the Gaussian white process. The model was experimentally confirmed by earthquake experiments, and the estimate of the maximum variance was used to estimate the standard deviation of the uncertainty at the time of sampling [9]. Ray et al. talked about the development, operation, and performance of intelligent flight sensors. The integrated microcontroller provides sensors with intelligent integrated sensor fault detection. An intelligent pressure sensor was introduced and tested in flight to increase reliability and ease of integration, leading to better data output [10]. Fabrizio et al. presented a mobile application on board and a portable electronic device. Sensors integrated into the electronics were used to collect data on passengers and cars. Usage data automatically adjust insurance coverage based on the car, environmental conditions, and preferences. The proposed solution could help reduce the costs of insurance changes and prevent insurance fraud [11]. Ranganathan and Smys proposed method used several smart sensors to detect damage to wind turbine structures. The sensors used in the proposed method estimate the damage index of the wind turbine with integrated software. The efficiency of the proposed method is measured by application to offshore wind turbines [12]. In this paper, embedded intelligent sensors are introduced to detect the effect of basketball teaching.

Before the experiment, the average scores of the experimental group and the control group in cross-quadrant jumping were 8.67 and 8.62, 6.42 and 6.35 in sitting and forward bending, and 8.14 and 8.02 in moving footsteps, respectively. There was no significant difference between the mean values of the test and control groups. After the experiment, the students' basic basketball skills were tested. The four test results of the control group were 65.36, 64.1, 65.43, and 65.16, respectively, and the improvement effect was not as good as that of the students in the experimental group.

## 2. Design Method of VR Basketball Teaching System

A system means that some parts constitute a whole. An extremely complex development object is called a system, which is composed of several components that interact and depend on each other to form an organic whole with specific functions [13]. This research is called the basketball system in order to achieve a certain goal in basketball education and achieve the mission of basketball education and teaching various forms of education and training. The basketball education system comprises four main components: teachers, students, educational content, and teaching aids. These four elements connect, interact, lock, and connect together and create a complex process of getting in and out of the system, and this is the basketball learning process. The functionality of the entire system is reflected in the results of the basketball process. There are six different relationships between the elements of the basketball teaching system [14]. As shown in Figure 1, it is the design mode of the basketball teaching system.

The selection of physical education course content should follow four basic principles: the characteristics of students' physical and mental development, the timeliness of the content, the interest, and the scientific nature of the content. When choosing physical education courses, it should be started from traditional, transforming existing, choosing life-oriented, and suitable teaching content for students to choose [15]. Attention should be paid to the selection of teaching content in the following aspects: the selected content should be in line with the teaching purpose. The selected teaching content should be in line with the students' personalities, interests, and hobbies. The selection of teaching content should be adapted to the region and season. An important task of physical education is to enable students to master certain sports skills in order to achieve fitness, enhance physical fitness, participate in competitions, and create achievements. Physical ability is acquired by learning, that is to say, physical ability is not innate but acquired. Learning inevitably involves a series of controls of cognition, memory, comprehension, application, and execution [16].

For present things, an understanding based on past experience and knowledge is needed so that the object of perception can be best explained and explained. The nature of this perception is called understanding. Different learning and understanding can affect the same things. Persistence of perception refers to the ability of the perceptual system to maintain a stable cognition of things in a specific area, and it will not change with the change of the environment.

Working memory can be maintained for several hours, during which time information is active and can be retrieved, that is, recalled. Through continuous repetition, working memory can retain meaningful information in the brain in the form of neural networks and can form connections with other retained information [17]. Memory starts from the perception of information, and it forms an instant memory from feeling. After preliminary processing, it enters a certain working state and becomes working memory. Both instantaneous memory and working memory are prone to forgetting and can only be stored as long-term memory through certain repetition and further refined processing. The content of long-term memory forms the experience of the individual and constitutes the cognitive belief system through gradual accumulation. The self-concept in the cognitive belief system, in turn, has a certain preference or inclination for the entry of information and information registration, selectively affecting the absorption of information [18].

Theoretical knowledge is a test of students' cognitive ability, and the evaluation of cognitive ability requires candidates to write some objective and subjective test questions to test students' understanding of teaching materials.

The brain is the central nervous system of the human body and is the physiological basis for learning. Each division of the brain has different functions, which both perform their own responsibilities and coordinate with each other. The main goal of basketball teaching is to improve basketball skills. Although basketball is a complex physical activity, it is always closely related to the control of the brain [19]. It can be seen from this point that in addition to strengthening students' physical quality and sports skills, basketball teaching should also focus on the cultivation of students' cognitive abilities such as thinking and imagination. In the teaching process, it is necessary to give students more self-control so that they can think actively and turn the teacher's experience into their own thoughts, so as to guide their own learning, rather than blindly relying on teaching. When students convert teachers' experiences into their own knowledge, knowledge needs to enter the students' long-term memory. When teaching, students should fully mobilize their senses, perceptions, attention, and so on and use multiple channels to simultaneously strengthen their understanding of the skills they have learned. On the one hand, basketball teaching cannot ignore the development of the brain. On the other hand, it is necessary to deeply understand the physiological mechanism of the brain to promote teaching and improve the teaching effect [20].  Figure 2 shows the cognitive model of motor skill formation.

Perception is very important in the formation of motor skills. When feeling the external environment, too much or too little sensory information may lead to wrong judgments. Perception is the mediator between the senses and the effector. Linking the two together, the correctness of the perception has a great impact on the learning of motor skills. Through practice, a series of motor schemas can be formed, that is, procedural memory is stored in long-term memory. These motor schemas are continuously consolidated, refined, and improved with practice. When developed to a certain level, they can achieve a highly coordinated automatic response without the need for feedback.

The law of effect states that learning occurs when there is an impact on the surrounding environment, that is, reinforcement after the reaction. Both reward and punishment reinforcement work on the incentive-response link.

Through the analysis of the essence of motor skills and the principles of learning and control, it can be seen that the typical closed skills are free throws, while most of the others belong to open motor skills. Different teaching methods should be adopted for different forms of motor skills to promote the rapid formation of skills. For open motor skills, in addition to teaching basic movements, it is also necessary to change the environmental background during practice, develop students' adaptability, promote the transfer of skills, and cultivate students' ability to use and innovate skills in different environments. Therefore, carrying out official competitions can provide a very good environment for students to use skills so that students can exercise and improve their skills in real competitions. The cognitive and control model theory of motor skills further embodies the role of the brain in motor skill learning. In the early stage of skill formation, the coordination between the brain and motor organs is not coordinated, and the control and participation of the brain to complete the action is relatively high. With the proficiency of the action, especially when it reaches the stage of automation, the brain is less involved in completing the action, and then people can free up space to shift their attention to other events. In the process of automatic action formation, feedback and reinforcement play a very important role. In the process of basketball teaching, teachers should pay attention to user feedback and reinforcement in order to speed up the formation and development of students' skills.

In basketball teaching, neither the teacher's teaching nor the student's learning can be ignored, but the time and methods of teaching and learning must be reasonably arranged. Each teacher has his own teaching philosophy, which is based on what kind of learning theory to focus on. Learning theories include behaviorism, cognitivism, and constructivism. Both behaviorism and early cognitivism are learning theories that emphasize behavioral responses, which can be called objectivism. The later cognitivism and constructivism emphasize the subjective initiative of the individual and believe that knowledge is constructed rather than taught by teachers, so it can be called constructivism. In basketball teaching, practice is essential. The theoretical basis of the guided practice should be objectivism, and the cognitive aspect should focus on the constructivist learning concept, which does not turn the improvement of students' abilities into the duplication of teachers' knowledge and experience. Students must have their own understanding and thinking in order to apply the skills acquired through practice to a greater extent.

According to the theory of item group training, basketball belongs to the skill-dominant category of same-court confrontational item groups. The confrontation in basketball is mainly manifested in the confrontation between offense and defense. Offense and defense exist at the same time and can be switched instantaneously. When one side is attacking, the other side is defending, and vice versa. Offense and defense can be switched quickly. Once the offensive side loses the ball, it must immediately switch to the defense. Once the defending side controls the ball, it will switch to the offense. Offense and defense are a pair of contradictory unity. It is reflected in the teaching that teachers should not only pay attention to offensive or defensive skills but ignore the other side of the contradiction. When teaching offensive skills, teachers can take into account the defense at the same time because only the technology that can break through the defense is an effective offensive technology.

At present, the teaching effect of the basketball teaching system is generally not good. For this reason, embedded intelligent sensors and VR technology are introduced in this paper. An embedded sensor is a sensor with a microprocessor, which is the product of the combination of a microcomputer and a sensor. The collected human-specific motion signal data will inevitably have interference and a certain zero drift. The purpose of preprocessing is to remove noise to prevent interference to useful signals and data and to restore signal and data degradation caused by factors such as circuit impedance matching. Preprocessing usually involves digital filtering and normalization. To identify the pattern, the sample data cannot be included directly in the classification for the activity classification because the sample data length is too long and the data size is too large. Therefore, it is necessary to construct a real estate space using the algorithm to generate the appropriate functions and introduce a limited dimension of the function in the classification for the classification and identification of functions. Feature extraction refers to a certain mapping of the feature space through a certain algorithm so that the dimension of the feature space changes from high to low. The features obtained after transformation are usually called secondary features; they are not any kind of original features and generally do not have physical meaning.

Usually, due to inertia, the motion of an object has a tendency to maintain its original motion state, so the most important part of a person's motion trajectory is the part where the motion state changes. To judge a person's action behavior, often the most representative things are the occurrence of stopping, accelerating, and changing direction. Human body motion signal refers to various dynamic information that changes with time during the operation of the human body and is picked up, recorded, and stored by various testing instruments. As shown in Figure 3, the embedded sensor and its application network for human action recognition are shown.

The following is the action recognition-related algorithm:

(1) $$\begin{array}{c} n=\frac{m-\text{Min}}{\text{Max}-\text{Min}},\\ n=\frac{\arctan\left(m\right)*2}{\pi }, \end{array}$$

where *m*– value before conversion and *n*– value after conversion.

(2) $$\begin{array}{c} II\left(t\right)=\sqrt{i_{m,t}^{2}+i_{n,t}^{2}+i_{z,t}^{2}}, \end{array}$$

where *II*(*t*)– velocity amplitude.

(3) $$\begin{array}{c} s_{u}\left(m\right)=\underset{v=1,2,\ldots ,B_{u}}{\min}m-n_{v}^{u},\\ a=\underset{u=1,22\ldots ,c}{\arg\min}\left(s_{u}\left(m\right)\right), \end{array}$$

where *m*– data to be tested and *s*_*u*_(*m*)– decision function.

(4) $$\begin{array}{c} M_{l}=\frac{1}{b}\overset{b}{\underset{v=1}{\sum }}M_{lv}, \end{array}$$

where *M*_*l*_– the maximum value of the amplitude at a certain time.

(5) $$\begin{array}{c} \bar{M}=\frac{1}{b}\sum_{u=1}^{b}\left|m_{u}\right|, \end{array}$$

where $\bar{M}$– average value after absolute value processing.

(6) $$\begin{array}{c} \varphi_{m}=\frac{{\left[\int_{-\infty }^{\infty }{\left|m\right|}^{p}l\left(m\right)\text{d}m\right]}^{1/p}}{{\left[\int_{-\infty }^{\infty }{\left|m\right|}^{a}l\left(m\right)\text{d}m\right]}^{1/a}}, \end{array}$$

where *l*(*m*)– probability density function.

(7) $$\begin{array}{c} \omega_{m}=\left\{\int_{-\infty }^{+\infty }{\left[m\left(t\right)-\bar{M}\right]}^{2}l\left(m\right)\text{d}m\right\}, \end{array}$$

where *ω*_*m*_– the standard deviation of the signal.

(8) $$\begin{array}{c} F=w\frac{av}{\Delta t}=ai\cdot q, \end{array}$$

where *F*– average reaction force.

(9) $$\begin{array}{c} AAI\left(t\right)=\frac{1}{b}\sum_{u=1}^{b}II\left(u\right), \end{array}$$

where *AAI*(*t*)– the mean value of the amplitude.

(10) $$\begin{array}{c} \left|II\left(u\right)-AII\left(k\right)\right|<Tg, \end{array}$$

where *Tg*– threshold.

(11) $$\begin{array}{c} \theta =\arcsin\frac{I\left(t-T_{1}\right)*I\left(t+T_{2}\right)}{II\left(t-T_{1}\right)\cdot II\left(t+T_{2}\right)},\\ M\left(t\right)=\tau \left(t-1,t\right)M\left(t-1\right)+\sigma \left(t-1\right), \end{array}$$

where *θ*– the included angle of the acceleration vector and*M*(*t*)– motion state quantity.

(12) $$\begin{array}{c} M\left(t\right)=\sum_{k=1}^{b}C\left(k\right),\\ \tau \left(t-1,t\right)={\left(A^{T}A\right)}^{-1}A^{T}Z, \end{array}$$

where *M*(*t*)– one-dimensional state quantity and *τ*(*t* − 1, *t*)– state transition value.

(13) $$\begin{array}{c} M\left(t\right)=M{}^{\prime }\left(t\right)+K{}^{\prime }\left(t\right)\left(N\left(t\right)-GM{}^{\prime }\left(t\right)\right),\\ L{}^{\prime }\left(t\right)=\tau \left(t-1,t\right)L\left(t-1\right)\tau {}^{\prime }\left(t-1,t\right)+W\left(t-1\right), \end{array}$$

where *M*(*t*)– posterior estimate and *L*′(*t*)– prior variance.

(14) $$\begin{array}{c} L\left(t\right)=\left(U-K\left(t\right)G\right)L{}^{\prime }\left(t\right),\\ K\left(t\right)=L{}^{\prime }\left(t\right)G^{T}\left(GL{}^{\prime }\left(t\right)G^{T}+R\left(t\right)\right), \end{array}$$

where *L*(*t*)– posterior variance and *K*(*t*)– gain at a certain time.

Virtual reality is a virtual object or environment that is created or simulated by computer technology and is similar to reality, including things and environments that are achievable, difficult to achieve, and impossible to achieve. Virtual reality technology is a new type of media technology, which includes performance technology, perception technology, interaction technology, and so on, while virtual reality is its media form, which can become a medium for conveying and transmitting content information.

The experiencer can manipulate elements in the virtual environment to a certain extent and can receive feedback from the environment in real time. In virtual reality, the phenomenon of human-computer interaction generally requires the help of virtual reality equipment such as helmet-mounted displays and gloves. Through these virtual reality devices, the information and clues felt in the real environment are transmitted to the experiencer through a variety of channels so that it produces a feeling of directly communicating and communicating with objects in the real environment. For example, the experiencer walks around in a virtual scene, and his sight changes with the movement of his body and head. When he grabs an object, his hand will feel like he is holding the object, and he can feel the weight of the object.

Compared with traditional teaching methods, virtual reality technology has obvious advantages and differences. It has many advantages and characteristics such as teaching virtualization, simulation, and remote control.

Presence refers to the sense of reality experienced by the experiencer as the protagonist in the virtual environment. In the virtual environment, the experiencer changes from a bystander to a participant. They not only can experience an immersive feeling but also can receive clues and information through various sensory organs such as smell, vision, hearing, and so on so that they are deeply immersed in it, resulting in a sense of immersion. When using virtual reality technology to provide new ideas and new ways to solve these problems, people should give full play to their creativity and imagination to give full play to the advantages and potential of virtual reality. When people experience the virtual environment, they can obtain both perceptual and rational knowledge, so as to obtain their own feelings and understanding of things. This acceptance is not passive but innovative and active.

Virtual reality can be suspended, and users can enter and exit the virtual world anytime, anywhere, as long as they have the relevant equipment. Virtual reality should be livable or at least have the potential to be livable. Multiple users can exist in the same space at the same time and can communicate with each other. Virtual reality is creative and should allow the experiencer to create objects or move freely. Through the use of wide area network promotion and development, virtual reality should not be limited to the location of the server but should be spread and promoted through the network, so as to become global.

Human-computer interaction in virtual reality is usually realized with the help of virtual reality devices such as helmets and gloves. Virtual reality, on the other hand, communicates everything it perceives to the user in a different way, just like in the real world.

In virtual reality, the virtual environment is the place where the experiencer lives, as well as the place where all activities and communication behaviors take place. The physical environment is the main component of the virtual environment. For example, the experiencers feel the difficulty of field practice in virtual reality and have a sense of fatigue, so they will be in awe and worry about field practice. Therefore, they may give high priority to the event. Adequate preparations should be made in advance of the event. It is also possible to make them feel intimidated and fearful. When making a virtual environment, in addition to setting the space of the virtual environment, the virtual environment should also be adjusted and repaired appropriately.

In the physical environment of the virtual world, experiencing a grueling experience creates a sense of fear and worry, which leads them to take the game seriously. In this game, they have to be well prepared to prevent them from feeling scared and uneasy.

Because there is indeterminacy in conventional teaching and learning practices, the intertemporal communication capability of virtual reality technology can well avoid such indeterminacy and help ensure the smooth and proper implementation of hands-on activities. In fact, the parallel multisensory channels of virtual reception can effectively enhance the immersion, presence, and reality experience that users get in the process of using them, effectively improving students' study experience and interest. Although virtual reality cannot fully replace traditional learning activities, it can help traditional learning activities and contribute to a certain extent to the normal development of coordination. As shown in Figure 4, it is the implementation framework of VR basketball teaching auxiliary training.

## 3. VR Basketball Teaching System Design Experiment

Two groups of voluntary students were selected and taught by coaches of the same level. The coaches had rich experience in basketball training. Most of the students in the experimental and control groups were inexperienced students. Their training period was one semester. In order to ensure the coherence of the experiment, the experimental group and the control group used the same field, basketball, and so on. After the training, relevant tests were carried out, and statistics were made. As shown in Figure 5, it is a flow chart of basketball training.

In order to exclude the interference of other factors and more accurately prove the auxiliary training effect of virtual reality technology, the homogeneity test of the experimental subjects was carried out before the experiment. The homogeneity test was divided into three parts: physical fitness, basketball learning experience, and sports interest. The test results are shown in Tables 1–3.

It can be seen that for the three physical condition tests, the means of the pilot and control groups, which were relatively frequent, did not differ much. This indicates no clear separation in fitness between the experimental and control groups. The respondents in the experimental and control groups were all novice basketball players. Their learning experiences are homogeneous.

The data to be sent by the embedded sensor is encapsulated in the frame format, and the data is sent to the buffer area of the sending data in the Ethernet chip over a long distance. Then an instruction is issued to realize the sending of the frame. As shown in Figure 6, it is the flow chart of the smart sensor for action recognition.

According to the action recognition process, the basic basketball quality of the students before the experiment was tested, as shown in Figure 7, which is the test results. In the one-minute fixed-point shooting test, the experimental class and the control class conducted independent sample tests. The shooting score was calculated by the number of shots in one minute, and the score in the fixed-point shooting in one minute was obtained. The average shooting scores of the experimental group and the control group were 2.64 and 2.83, respectively, and the passing and receiving scores were 8.12 and 8.01, respectively. It can be seen from Figure 7 that there is no significant difference between the experimental class and the control class in the test.

In the exercise load measurement of the experimental group and the control group, the heartbeat frequency was used as a reference to indirectly reflect the different physical loads of the two groups during the exercise process. The test results are shown in Figure 8.

The mean heart rate in the 4 sports of the experimental group was 145, 130, 155, and 120, respectively, higher than that of the control class. In sports practice, the greater the physical load within the safe load limit for cardiac work is, the more comfortable the physical development of the students will be. However, the working load of the experimental class is much higher than that of the control class.

After the experiment, the basic physical fitness data of the two classes after the experiment were compared to compare the differences between the students in the two classes. The comparison results are shown in Figure 9.

The test data in Figure 9 was compared with the physical fitness of the students before the experiment. In the four tests, the interest enthusiasm of the students in the experimental group made the students fully devote themselves to the daily teaching training. This ensures that each part of the student's body can exercise with a large load. The scores of the experimental group on the four test items were 11.36, 9.557, 1.87, and 8.17, which were higher than those before the experiment. Their physical fitness was greatly improved.

After the experiment, a comparative analysis of the basic basketball skills tests data information of the two classes after the experiment was made.  Figure 10 shows the test results.

As can be seen from Figure 10, in the four basketball skill tests, the experimental group performed better than the control group. It can be found that the virtual reality teaching method designed in this paper has certain advantages over the traditional basketball teaching method, which can stimulate students' learning motivation and strengthen their participation. Each student can participate and practice well, and the students can improve their basic basketball skills in a pleasant and cheerful environment.

## 4. Conclusions

In the environment of industrial informatization, the use of virtual reality technology in basketball teaching is of great significance for cultivating students' interest in basketball and cultivating students' autonomy and exploration. The most representative features of human motion and behavior are stopping, accelerating, and changing direction. The effective teaching of basketball relies on teachers' understanding of students' interests, motivation, emotions, physical fitness, technology, tactics, and other aspects, so as to clarify students' actual learning goals and carry out targeted teaching to achieve the goals. According to the characteristics of basketball, an embedded sensor for action recognition is designed, and its application in sports training is verified. In the test data of basic basketball skills after training, the experimental group was significantly higher than the control group, and there were significant differences in the test data, indicating that virtual reality technology-assisted training is of great help to the improvement of basic basketball skills. This paper makes a preliminary prediction, but due to the limitations of data sources and academic standards, some omissions inevitably appear in this paper. The analysis in the status analysis stage is not comprehensive, only showing the changes of relevant indicators and lacking the analysis of the internal judgment. Theoretically, it has not yet been fully grasped. This paper puts forward some suggestions and strategies for the application of virtual reality technology in education. The feasibility and operation steps of these suggestions and strategies still need to be tested in practice.

## Figures and Tables

**Figure 1:** Design pattern of basketball teaching system.

**Figure 2:** Cognitive models of motor skill formation.

**Figure 3:** Human action recognition embedded sensor and its application network.

**Figure 4:** VR-assisted training implementation framework.

**Figure 5:** Basketball experimental training flow chart.

**Figure 6:** Smart sensor software flow chart.

**Figure 7:** Basic basketball quality of students.

**Figure 8:** Heart rate test results.

**Figure 9:** Postexperimental physical fundamentals.

**Figure 10:** Basic basketball technical test data after the experiment.

**Table 1:** Physical fitness test results.

	Standing long jump (cm)	30s jump rope (times)	Basketball throwing long (m)
Experimental group	128.84 ± 13.38	44.36 ± 7.3	3.43 ± 0.35
Control group	127.81 ± 17.42	41.75 ± 7.31	3.23 ± 0.43
T	−1.235	−1.67	0.618

**Table 2:** Learning experience.

	More than 3 months of study experience		Learning experience within 3 months		Never been exposed to	
	Number of people	Percentage (%)	Number of people	Percentage (%)	Number of people	Percentage (%)
Experimental group	2	6.67	2	6.67	26	86.67
Control group	3	10	2	6.67	25	83.3
Total	5	8.33	4	6.67	51	85

**Table 3:** Basic physical fitness.

Test content	Experimental group	Control group	*P*-value
Cross-quadrant jump	8.67 ± 3.35	8.62 ± 3.57	0.12
Sitting forward bend	6.42 ± 4.81	6.35 ± 7.62	0.47
Foot movement	8.14 ± 0.36	8.02 ± 0.54	0.17

## Data Availability

The data used to support the findings of this study are available from the corresponding author upon request.
